# Socioeconomic Influence on Cardiac Mortality in the South Asian Region: New Perspectives from Grey Modeling and G-TOPSIS

**DOI:** 10.1155/2021/6866246

**Published:** 2021-11-10

**Authors:** Shazia Rehman, Erum Rehman, Iftikhar Hussain, Zhang Jianglin

**Affiliations:** ^1^Department of Dermatology, Shenzhen People's Hospital, The Second Clinical Medical College, Jinan University, The First Affiliated Hospital, Southern University of Science and Technology, Shenzhen 518020, Guangdong, China; ^2^Candidate Branch of National Clinical Research Center for Skin Diseases, Shenzhen, China; ^3^Department of Biomedical Sciences, Pak-Austria Fachhochschule, Institute of Applied Sciences and Technology, Haripur, Pakistan; ^4^School of Economics, Shandong University of Finance and Economics, Jinan, China; ^5^Department of Mathematical Sciences, Karakoram International University, Gilgit, Pakistan

## Abstract

**Background:**

Measuring the potential socioeconomic factors of cardiac mortality is fundamental to identifying treatments, setting priorities, and effectively allocating resources to minimize disease burden. The study sought to present a methodology that explores the connections between urbanization, population growth, human development index (HDI), access to energy, unemployment, and cardiovascular disease (CVD) mortality within the South Asian Association for Regional Cooperation (SAARC) nations to mitigate the cardiac disease burden.

**Methods:**

This investigation uses multiple-criteria decision-making methodologies to analyze data between 2001 and 2017 commencing with a mathematical grey incidence analysis (GIA) methodology to estimate weights and rank nations based on CVD mortality. Then, utilizing the conservative min-max model approach, we sought to determine which country contributes the most to CVD mortality among all South Asian nations. The grey preference by similarity to ideal solution (G-TOPSIS) method is adopted for further optimization by prioritizing the selected factors that have the greatest influence on CVD mortality.

**Results:**

The estimated statistic highlights that, among SAARC nations, Pakistan has a significant proportion of the disease burden attributable to cardiac events. In addition, HDI showed a significant contribution in the reduction of CVD mortality, whereas unemployment showed a significant contribution in the rise of CVD mortality among all selected variables.

**Conclusions:**

This investigation may facilitate researchers with a multiple-criteria decision-making roadmap to help them enhance the quality of their studies and their understanding of how to use multiple-criteria decision-making techniques to evaluate and prioritize the influencing factors of disease mortality in healthcare research. Further, the study outcomes provide additional practical knowledge for appropriate policy solutions.

## 1. Introduction

Cardiovascular diseases (CVDs) are the world's leading cause of death and disability [1]. CVD-related deaths have declined in several high-income countries (HICs) during the last several decades but have grown in low- and middle-income countries (LMICs), with about 80% of the burden falling on these nations [2, 3]. The population of South Asian nations has become 1.8 billion in 2020, accounting for 23% of the global population [4]. Chronic NCDs, especially CVD, are becoming a serious threat in LMICs, including the densely populated South Asian nations, as a result of fast industrialization, higher survival from acute diseases, and population aging [5]. NCDs now account for 52 percent of mortality in South Asia, and by 2030, they are expected to account for 72 percent of overall mortality [6, 7]. An abundance of evidence has shown that South Asians are at elevated risk of CVDs bringing about calls to upgrade CVD prevention in South Asian nations and migrant populations. CVD is a life-threatening, resource-intensive disorder that causes early death, disability, altered functional capability, reduced life quality, and the requirement for additional pharmacotherapies. In many economies, CVD is also a leading cause of hospitalization and healthcare spending [8, 9]. As a result, it poses a serious threat to patients, healthcare systems, and communities, primarily in countries with limited resources and economies. In this perspective, recent research suggests that South Asians may be at an elevated risk of CVD, which may present 10 to 15 years earlier in life in South Asians than in other geographic and ethnic/racial communities. These characteristics along with other structural difficulties have posed a significant challenge to the natural environment for healthy livings, contributing to a rise in disease burden, notably CVDs, and, as a result, causing significant economic repercussions [10]. Understanding the variables that cause CVD-related mortality is fundamental to identifying treatments, setting priorities, and effectively allocating resources to minimize disease burden. Reporting the consistency or differences in the relationships between CV-associated factors and mortality, both worldwide and country-wise grouped by monetary levels, would aid in the establishment of global and context-specific prevention measures. Furthermore, there is a literature gap that might contribute to and advance our understanding of CVDs in terms of socioeconomic factors. Evaluation outcomes from a broader disease perspective represent the adaptability of healthcare systems in an economy and function as a useful reference point.

Multicriteria decision analysis (MCDA) methodologies were acquainted within the healthcare domain as a proper decision‐support strategy for dealing with complex issues via convenient approaches [11]. These methodologies were likewise used to assist decision makers with criteria evaluations for comparisons, to support health technology assessment decision‐making processes and regulatory decisions during pandemic influenza, to evaluate the quality of care and screening needs, characterize new medical equipment plans, define new fee schedules, compare methods for the suitability, assess potential harms, select healthcare waste treatment technologies, enhance outpatient services, support early diagnosis, select an infrastructure's localization, optimize a process, and evaluate the quality of medical devices. These techniques are regarded for a variety of reasons. Researchers believed that the procedure allows visibility, consistency, and precision toward a more reasonable priority setting from a methodological standpoint [12, 13] . In a broader sense, the MCDA application procedure is regarded as efficient and successful in healthcare settings.

The issue of multiple objectives often exists in the problems within systems, increasing the ambiguity of decisions. In this setting, to minimize errors, it is significant to find techniques that include the greatest number of criteria in the decision-making process that direct influence decisions [14, 15]. However, most of the time this technique is difficult to execute, because, in many cases, the decision-making criteria vary, raising the degree of uncertainty of the final response. These procedures are much more complicated in the field of health, as they include not only technological or economic problems but also the human element, which creates conflicts of interest and hinders the final decision. Hence, several types of research are performed using MCDA to improve health systems as a whole [16]. These researches have been conducted using various techniques to explore the relationship between CVD mortality and associated factors. However, knowledge regarding the best approaches to enhance the quality of research work and its implementation is sparse. In the present investigation, we integrated grey modeling with MCDA approaches to seek a comprehensive understanding of CVD mortality and associated factors across SAARC nations. However, by addressing all SAARC nations together with a wide range of factors, we may provide a more dynamic spectrum of the interactions. In response, the present study attempts to bridge the existing literature gaps by exploring the tie between urbanization, population growth, HDI, access to energy, unemployment, public health expenditure, and CVD mortality of SAARC nations (Pakistan, Bangladesh, Maldives, Afghanistan, Nepal, India, Sri Lanka, and Bhutan). To explore this association, we deployed mathematical GIA modeling of grey system theory (GST) which comprised of Deng degree of GIA, absolute degree of GIA, and the second synthetic degree of GIA. In addition, this study utilized the conservative (min-max) criteria and grey TOPSIS to conduct a comparative analysis of all the selected factors and CVD mortality among SAARC nations to ascertain which country and the related factors contributing more to mortality. The schematic diagram of the study is presented in Figure 1.

## 2. Materials and Methods

### 2.1. Data Source

For the period 2001–2017, information on the variables (urbanization, HDI, access to energy, unemployment, public health expenditure, and CVD mortality in the SAARC nations (Pakistan, Bangladesh, Maldives, Afghanistan, Nepal, India, Sri Lanka, and Bhutan)) are abstracted from Our World in Data. We used publicly available data; therefore, we will not be making that available.

### 2.2. Grey Incidence Analysis (GIA) Method

GIA models, often defined as models of the grey relational analysis (GRA), are considered an early aspect of the new grey system theory (GST) [17]. The GST was founded on remarkable work done in 1982 by a Chinese scientist, named Professor Julong Deng, and has been employed in different domains of learning since that time for dealing with vulnerability problems caused by insufficient information and mostly unclear processes. Professor Deng acquainted the notion of the grey relational grade (GRG) to GIA's model in 1985 [17]. The GIA model is proven to be superior to other statistical models of systems analysis [18]. The GST is designed to bridge the gap between the natural and social sciences. The degree of data transparency is used to designate GST. GIA approaches establish one of the key subjects of GST to deal with ambiguous systems with limited information. GST has a place with the group of uncertainty theories, which also includes rough set theory, interval theory, fuzzy theory, and so on. Nonetheless, GST directed through its unique methodologies handles vulnerability differently from other vulnerability speculations. GST classifies the world's systems into three categories: white, black, and grey. A black structure refers to one in which no data is provided, whereas a white structure refers to one in which complete information is accessible. Thus, a GS turns into a framework with incompletely known and somewhat obscure data. GST and its models are known for their ability to anticipate and make decisions based on small sample sizes, erroneous and insufficient information [19, 20]. The GIA models endeavor to comprehend ambiguous relationships between the characteristics inherent with GST. The fundamental concept of GIA is that the degree of closeness (correlation) of the geometrical structure of the data series indicating the structure variables may be used to anticipate the closeness of a relationship between the system variables. In the literature, this closeness is referred to as proximity. Deng's degree of GIA, absolute degree of GIA, and second synthetic degree of GIA are the three components of the GIA model. In essence, the D-GIA model measures the influence of one variable indicated by a data set exerts on the other, while the A-GIA model measures the association (integral proximity) between the two [21, 22]. Furthermore, the second synthetic GIA model provides an estimate of an overall measure of association between the parameters under investigation. The algorithms involved in the computations of GIA are summarized in Figure 2. The detailed description of GIA models can be read in Liu et al.[23].

The data are analyzed by employing GIA methods (Deng DGIA, absolute DGIA, and SSD-GIA). These models are designed using SPSS (v26, IBM, United States) and Microsoft Excel (2019) software. The conservative (min-max) approach is adopted for decision making under uncertainties [24]. Additionally, grey TOPSIS methodology is employed to hierarchize the selected factors that have a greater impact on CVD mortality within the South Asian region [25].

## 3. Results and Discussion

The present investigation is carried out using grey incidence approaches to quantify the strength of association between socioeconomic variables and CVD mortality among SAARC countries over the period 2001–2017.  Table 1demonstrates the outcomes of grey incidence models, namely, Deng D-GIA, absolute D-GIA, and SSD-GIA for CVD mortality and associated factors among SAARC countries. The absolute D-GIA and the SSD-GIA models have values ranging from zero to one, whereas Deng GRG has values ranging from 0.5 to 1. It is also considered highly associated if it is near to 1 and weak if it diverges from 1. For the sake of clarity, the ranking sequences based on GIA are displayed in Table 2in decreasing order. The graphical representation of the association among chosen variables based on GIA findings is displayed in Figure 2.

 
*Urbanization.* According to GIA findings, Pakistan has the highest linkage between urbanization and CVD-related mortality, whereas the weakest association is observed for the Maldives, and both countries sustained their position under all grey incidence models. After Pakistan, Bhutan acquired the highest weight trailed by Bangladesh and Nepal. Altogether, the estimates from the SSD-GIA model uncover that, among South Asian economies, Pakistan had all the earmarks of being the main country where urbanization is observed highly associated with CVD mortality in its populace. In South Asia, Pakistan has the most elevated pace of urbanization. As per United Nations Population Division evaluations, over half of the country's population will be living in cities by 2025. Many emerging nations have experienced urbanization without development, employment, or productivity. Only effective public policies can reap the benefits of urbanization. Slum-dwellers, environmental pollution, poor health consequences, poverty, and disparity have all emerged from unplanned and uncontrolled urbanization. Pakistan, too, is dealing with a slew of urban issues [26].
 
*Population Growth.* Many studies demonstrate that population growth is consistently and firmly linked to an elevated risk of CVD incidence and fatalities across the globe [27, 28]. According to the findings, Sri Lanka, Bhutan, Maldives, Pakistan, India, and Bangladesh sustained their ranking position under all GIA models. The strength of closeness is seen higher in the case of Sri Lanka trailed by Bhutan, implying that the population growth of Sri Lanka is closely and positively associated with mortality of CVD in its population. The findings back up prior investigations substantiating the relationship and significance of population growth in the development and progression of CV disorders [29, 30].
 
*HDI.* As per GIA findings, the ranking order appears to be the same for Pakistan, indicating a strong positive linkage of CVD mortality and HDI in its population led by Afghanistan among the SAARC region. The significant linkage between CVD deaths and HDI in Pakistan demonstrates the most noteworthy factor for evaluating and foreseeing CVD mortality. Among the SAARC region, the Maldives and Sri Lanka showed up with the least grey incidence weights, indicating the weakest relationship of HDI with CVD-related mortality against all grey models. Among all SAARC nations, the most fragile association is seen in the population of Sri Lanka, which indicates that HDI is a predictive factor to assess and predict cardiac events. The HDI is a social and monetary indicator of economies worldwide and could be linked to a variety of illnesses, including CVDs. The present findings corroborate dozens of prior studies that show a substantial role of HDI in the population's health and mortality [31, 32].
 
*Access to Energy.* Considering the effect of access to energy on CVD mortality among SAARC region, Pakistan, Sri Lanka, Bhutan, Bangladesh, India, and Afghanistan sustained their positions against all grey models; however, the strength of association is determined to be stronger for Pakistan than the rest of the countries. Nepal and Maldives positioned 4^th^ and 5^th^ under DD-GIA and SSD-GIA models, respectively, yet shuffled their position against the AD-GIA model. More precisely, the factor access to energy had all the earmarks of being more striking on CVD deaths in the populace of Afghanistan. The findings exhibited that access to energy is a vital element to evaluate and anticipate deaths from cardiac events in the inhabitants of Afghanistan. According to the estimated GIA result, SAARC nations generated energy using gasses and nonrenewable fuel means without considering the environmental and public health consequences. The breadth of epidemiological research is consistent with the current study's findings depicting a substantial linkage between atmospheric pollution from energy use consumption and a range of CV disorders and related mortality [33].
 
*Unemployment.* Unemployment is a considerable cause of mortality and morbidity, particularly especially if it lasts for a long duration. An investigation by Méjean et al. exhibited a 20% rise in the risk of coronary heart disease events in an unemployed French populace without prior coronary illness [34]. At an aggregate level, unemployment appeared to be a substantial factor of cardiac mortality in the Indian populace and ranked top based on findings of DD-GIA and SSD-GIA models with comparatively higher strength of association. Sri Lanka and Bangladesh ranked second and third, respectively, among all.
 
*SAARC Nations*. Maldives and Nepal showed the least amount of weights assessed by AD-GIA and the SSD-GIA models, which implies that these nations reflect the least share of disease burden across South Asian nations owing to unemployment. India is the world's second most populous country and the first among the SAARC nations. Despite the government's endeavors, India continues to be a country with significant unemployment issues [35, 36]. The substantial connection between unemployment and cardiac mortality in the Indian population recommends that there is a pressing requirement for improved employment opportunities to minimize the disease burden.
 
*Public Health Expenditure.*Table 1 shows a review of the relationship between public health expenditure and cardiac mortality in South Asian nations using GIA models. The outcomes of this study reinforce earlier investigations substantiating the relationship and significance of public health expenditure with CVD-related disorders and mortality. Given the weights determined for each of the three GIA models, India, Bangladesh, Maldives, and Bhutan maintained their position and ranked first, second, third, fourth, seventh, and eighth, respectively. Notwithstanding, Maldives and Bhutan are regarded as the less significant nations when it comes to the influence of public health expenditure on cardiac mortality among South Asian countries. Surprisingly, Bhutan appeared to be on the top among all South Asian nations, where a most fragile association is seen between cardiac mortality and public health expenditure. The study backs up earlier researches that, in emerging nations with low per capita incomes, an indiscriminate rise in government health spending with a high opportunity cost might negatively impact the population's health. The conceivable justification for this peculiarity can be that the marginal benefit of higher government spending is less than the marginal cost of additional taxes. The outcomes presented in the present study focuses on the way that increment in government spending alone might be insufficient to attain the ideal improvements in cardiac health outcomes. These findings corroborate with prior research that increasing public health spending does not guarantee improved health outcomes [37, 38].

For a comparative decision analysis, a decision-making strategy must be constructed before it can be used. The SSD-GIA between the decision actions (*F*_*k*_) and decision criteria (*C*_*p*_) are reported in Table 3, which is based on the SSD-GIA based matrix. Here, we have *k* = 6, *p* = 8, and output = *v* (*A*_*k*_, *C*_*p*_), whereas *k* = 1, 2, 3, 4, 5, 6 and *p* = 1, 2, 3, 4, 5, 6, 7, 8. The definition of decision parameters is elaborated in Table 4.

### 3.1. The Conservative (Min-Max) Criterion

We, then, utilized the conservative min-max approach based on the estimated results of SSD-GIA to distinguish which country is contributing more to raising CVD mortality among South Asian economies against the selected factors. This criterion was implemented in accordance with instructions used in Prasad [39] and Rehman et al. [24]. Since CVD mortality is to be minimized, a min-max criterion is embraced as shown

(1) $$\begin{array}{c} \min C_{p}\left\{\max F_{k}v\left(F_{k},C_{p}\right)\right\}=\min C_{p}\left\{\begin{array}{c} 0.85005\\ 0.86363\\ 0.85508\\ 0.85007\\ 0.85347\\ 0.90057\\ 0.90210\\ 0.85891 \end{array}\right\}\\ =0.85005. \end{array}$$

For the chosen parameters in the study, the estimated statistics demonstrate that Pakistan has a significant proportion of the illness burden owing to cardiac events among the SAARC nations. Pakistan is one of the world's most populated countries, having the greatest population growth rate in South Asia at 2.40 percent. As the nation develops economically, the behavioral changes of the populace have culminated in a shift in the population's health profile. In addition, for the past few decades, Pakistan has spent less than 1% of its gross domestic product (GDP) on population health, despite the World Health Organization's (WHO) recommendation of at least 6% of the GDP for health spending [40, 41]. The output of the decision-making approach highlights the fact that Pakistan has the potential to foster a new strategy and take remedial measures to reduce the overall CVD mortality in the South Asian region. Presently, the query is among the chosen variables which have the greatest impact on the ascent of CVD mortality across all South Asian nations. We utilized the grey TOSIS technique to gain this additional insight.

### 3.2. Grey TOPSIS Analysis

In this section, we adopted grey TOPSIS to estimate and rank the strength of the six explanatory variables (urbanization, population growth, HDI, access to energy, unemployment, and public health expenditure) on cardiac mortality for each country in the SAARC region. Using linguistic variables, we converted the decision-making criteria into grey numbers and then created a weighted normalized grey decision-making matrix for each of the explanatory variables across all South Asian nations independently. Based on that, we determined the patterns for the ideal (*F*^max^) and anti-ideal (*F*^min^) solutions and then computed the distances of the alternatives (*F*_1_–*F*_6_). In doing so, access to energy, HDI, and public health expenditure is regarded as benefit criteria, whereas unemployment, urbanization, and population growth are considered nonbenefit criteria.  Table 5 displays the ideal and anti-ideal solution results, while Table 6 shows the estimated intervals from the ideal (*F*^max^) and anti-ideal (*F*^min^) solutions.

Further, we computed the grey synthetic assessment degree of the specified alternatives based on the distances (**D**^**+**^,**D**^−^) determined in Table 6: *F*_1_ = 0.463, *F*_2_ = 0.295, *F*_3_ = 0.723, *F*_4_ = 0.509, *F*_5_ = 0.275, and *F*_6_ = 0.545. Then, we generated a descending order rating of the alternatives as follows:

HDI > public health expenditure > access to energy > urbanization > population growth > unemployment.

In accordance with an elucidation of the grey TOPSIS synthetic assessment, it is concluded that HDI (0.723) contributes emphatically in diminishing CVD deaths among the selected variables in the SAARC region trailed by public health expenditure (0.545) and access to energy (0.509), while the unemployment (0.275) variable had all the earmarks of being the worst one in raising CVD mortality led by population growth (0.295) and urbanization (0.463) (Figure 3). Utilizing the MCDA techniques in the present study will assist the public health practitioners and policymakers in drawing decisions on the best way to minimize CVD mortality in the SAARC region by emphasizing the worse variables.

## 4. Conclusions

The outcomes of the analyses revealed that all the selected factors sway cardiac mortality in the South Asian nations with varying degrees of influence. To be more specific, our findings highlight the importance of planned urbanization, sustainable population growth, improved employment opportunities, adaptation of clean and renewable energy sources, raising the educational level, upgrading living standards, rapid access to quality health services, and public health expenditure investment in reducing cardiac risk. These contributing variables join into a progression of pathways that lead to various forms of CVDs [42–44].

Given the findings, this study concludes that HDI and unemployment are significant areas of concern for overall CVD mortality reduction in the SAARC region. Further investing in HDI and concentrating on employment opportunities may assist these economies to address the issue of CVD mortality. All the outcomes of the analyses are well-calibrated, and we may give experiences to the entirety of the characterized objectives of the investigation. Our findings have significant ramifications for public health policy and decision makers in terms of the sustainable development goals (SDGs) of good health and well-being (SDG 3), decent work and economic growth (SDG 8), sustainable cities and communities (SDG 11), affordable and clean energy (SDG 7), quality education (SDG 4), and partnerships for the goals (SDG 14). We must realize that the health sector is simply one of many factors to a healthy life expectancy to achieve a health objective with a CVD focus. Agriculture, environmental, transportation, and economic policies, along with international trade pacts, will all influence diet, physical inactivity, environmental sustainability, and access to better health facilities. We must work together and collaborate across regions and disciplines to promote and assert a significant return of interest in cardiac health; only then we will be able to persuade economies and businesses to contribute critical resources to our mutual goals, which is fundamental to population health and wellness among SAARC economies. Eventually, the governments in the SAARC nations should unanimously collaborate, encourage, and concentrate on strategies that can minimize the regional burden of CVD through planned urbanization, sustainable population growth, improvement in employment opportunities, adoption of clean and renewable energy sources, raising the educational level, enhancing living standards, improving access to quality health services, and investment in public health expenditure to mitigate the risk of CVD.

Researchers have agreed that the MCDA paradigm is productive in healthcare domains and is a beneficial decision‐making tool since it enables transparency, robustness, and consistency in the context of diverse and contradictory parameters [12, 45]. The study outcomes recommend that when confronted with various alternatives of equivalent worth in healthcare decision-making situations, researchers should employ MCDA methodologies and tools. This investigation may facilitate researchers with a multimethod roadmap to help them enhance the quality of their studies and their understanding of how to use multimethod techniques to evaluate and prioritize the influencing factors of disease mortality in healthcare research. Such investigations could assist improving our capacity to acquire valuable insights into the multifaceted nature of the variables in a system. Further, the suggested methodologies provide a valuable tool and additional practical knowledge for policy and decision makers in drawing rational decisions. However, further investigations are necessary to contrast the particularities of MCDA approaches (e.g., preferred inferencing approaches) and enable researchers in selecting the appropriate tool, as there is no rationale for why one MCDA technique is adopted over the other.

## Figures and Tables

**Figure 1:** The graphical abstract.

**Figure 2:** Grey comparative assessment of the selected parameters with CVD mortality.

**Figure 3:** Grey synthetic assessment degree for the selected explanatory variables.

**Table 1:** GIA assessment between CVD mortality and associated factors among SAARC nations.

SAARC nations	AD-GIA	DD-GIA	SSD-GIA
CVD mortality and urbanization			
Pakistan	0.87375	0.84687	0.86031
Bangladesh	0.87066	0.84049	0.85558
Maldives	0.65430	0.59470	0.62450
Afghanistan	0.79400	0.63250	0.71325
Nepal	0.86190	0.84497	0.85347
India	0.80245	0.77141	0.78693
Sri Lanka	0.81105	0.79009	0.80057
Bhutan	0.86823	0.85103	0.85963

CVD mortality and population growth			
Pakistan	0.82650	0.71666	0.77158
Bangladesh	0.68830	0.62008	0.65419
Maldives	0.85553	0.85463	0.85508
Afghanistan	0.71475	0.69743	0.70609
Nepal	0.75313	0.64587	0.69950
India	0.80301	0.70099	0.75200
Sri Lanka	0.90675	0.89745	0.90210
Bhutan	0.90537	0.81245	0.85891

CVD mortality and HDI			
Pakistan	0.85553	0.85463	0.85005
Bangladesh	0.81113	0.74103	0.77608
Maldives	0.62390	0.59880	0.61135
Afghanistan	0.88526	0.81476	0.85001
Nepal	0.76514	0.70098	0.73306
India	0.80374	0.79906	0.80140
Sri Lanka	0.61047	0.54369	0.57708
Bhutan	0.76115	0.63845	0.69980

CVD mortality and access to energy			
Pakistan	0.88981	0.85005	0.86993
Bangladesh	0.79610	0.76610	0.78110
Maldives	0.82483	0.77333	0.79908
Afghanistan	0.73696	0.68696	0.71196
Nepal	0.80117	0.79977	0.80047
India	0.78159	0.71239	0.74699
Sri Lanka	0.85886	0.84128	0.85007
Bhutan	0.85225	0.81291	0.83258

CVD mortality and unemployment			
Pakistan	0.83824	0.78990	0.81407
Bangladesh	0.88259	0.84467	0.86363
Maldives	0.73609	0.65473	0.69541
Afghanistan	0.81723	0.75009	0.78366
Nepal	0.72285	0.69993	0.71139
India	0.90180	0.89934	0.90057
Sri Lanka	0.90916	0.86730	0.88823
Bhutan	0.72846	0.73654	0.73250

CVD mortality and public health expenditure			
Pakistan	0.91079	0.84339	0.87709
Bangladesh	0.87679	0.83269	0.85474
Maldives	0.81736	0.71650	0.76693
Afghanistan	0.82849	0.79245	0.81047
Nepal	0.83660	0.74300	0.78980
India	0.93063	0.84783	0.88923
Sri Lanka	0.86548	0.81458	0.84003
Bhutan	0.74542	0.65472	0.70007

**Table 2:** Ranking based on grey incidence analysis.

Explanatory variables	SSD-GIA-based ranking order
Urbanization	Pakistan > Bhutan > Bangladesh > Nepal > Sri Lanka > India > Afghanistan > Maldives
Population growth	Sri Lanka > Bhutan > Maldives > Pakistan > India > Afghanistan > Nepal > Bangladesh
HDI	Pakistan > Afghanistan > India > Bangladesh > Nepal > Bhutan > Maldives > Sri Lanka
Access to energy	Pakistan > Sri Lanka > Bhutan > Nepal > Maldives > Bangladesh > India > Afghanistan
Unemployment	India > Sri Lanka > Bangladesh > Pakistan > Afghanistan > Bhutan > Nepal > Maldives
Public health expenditure	India > Pakistan > Bangladesh > Sri Lanka > Afghanistan > Nepal > Maldives > Bhutan

**Table 3:** Grey decision matrix.

SSD-GIA	C_1_	C_2_	C_3_	C_4_	C_5_	C_6_	C_7_	C_8_
F_1_	0.86031	0.83546	0.62450	0.71325	0.85347	0.78693	0.80057	0.84463
F_2_	0.77158	0.65419	0.85508	0.70609	0.69950	0.75200	0.90210	0.85891
F_3_	0.85005	0.77608	0.61135	0.85007	0.73306	0.80140	0.57708	0.69980
F_4_	0.86993	0.78110	0.79908	0.71196	0.80047	0.74699	0.85007	0.83258
F_5_	0.81407	0.86363	0.69541	0.78366	0.71139	0.90057	0.88823	0.73250
F_6_	0.87709	0.85474	0.76693	0.81047	0.78980	0.88923	0.84003	0.70007

**Table 4:** Definition of the decision parameters.

Parameters	Evaluating grey relational association between CVD mortality and associated factors among SAARC countries
SAARC countries (C_p_); p = 1, 2, 3, 4, 5, 6, 7, 8	Pakistan (C_1_)
	Bangladesh (C_2_)
	Maldives (C_3_)
	Afghanistan (C_4_)
	Nepal (C_5_)
	India (C_6_)
	Sri Lanka (C_7_)
	Bhutan (C_8_)

Explanatory variables (F_k_); k = 1, 2, 3, 4, 5, 6	Urbanization (F_1_)
	Population growth (F_2_)
	HDI (F_3_)
	Access to energy (F_4_)
	Unemployment (F_5_)
	Public health expenditure (F_6_)

**Table 5:** Ideal and anti-ideal solutions.

	C_1_	C_2_	C_3_	C_4_	C_5_	C_6_	C_7_	C_8_
*F* ^max^	[0.55, 0.65]	[0.42, 0.67]	[0.54, 0.88]	[0.40, 0.65]	[0.42, 0.60]	[0.55 ,0.91]	[0.52, 0.86]	[0.45, 0.77]
*F* ^min^	[0.23, 0.25]	[0.18, 0.34]	[0.20, 0.43]	[0.10, 0.15]	[0.17, 0.15]	[0.26, 0.56]	[0.20, 0.46]	[0.16, 0.17]

**Table 6:** Estimated distances of the alternatives (*F*_k_) from the ideal and anti-ideal solution.

	C_1_	C_2_	C_3_	C_4_	C_5_	C_6_	C_7_	C_8_
**D** ^+^								
F_1_	0.23	0.09	0.32	0.05	0.14	0.00	0.00	0.39
F_2_	0.00	0.23	0.18	0.40	0.28	0.32	0.36	0.19
F_3_	0.00	0.27	0.07	0.03	0.11	0.12	0.18	0.00
F_4_	0.31	0.00	0.34	0.04	0.28	0.00	0.11	0.06
F_5_	0.28	0.27	0.14	0.00	0.13	0.23	0.28	0.12
F_6_	0.12	0.21	0.24	0.00	0.23	0.00	0.12	0.19

**D** ^−^								
F_1_	0.14	0.20	0.08	0.35	0.01	0.12	0.15	0.00
F_2_	0.36	0.06	0.22	0.00	0.12	0.06	0.00	0.00
F_3_	0.36	0.02	0.33	0.38	0.00	0.00	0.16	0.13
F_4_	0.04	0.29	0.06	0.36	0.00	0.24	0.00	0.19
F_5_	0.14	0.02	0.13	0.12	0.00	0.03	0.11	0.00
F_6_	0.24	0.16	0.17	0.06	0.19	0.00	0.30	0.21

## Data Availability

The data used in the current study are publicly available at www.ourworldindata.org.
